This article has been retracted.

# Internet of Things Device Identification Algorithm considering User Privacy

**DOI:** 10.1155/2022/6173185

**Published:** 2022-04-25

**Authors:** Lin Wang

**Affiliations:** College of Physics and Engineering Technology, Chengdu Normal College, ChengDu, Sichuan, China

## Abstract

The Internet of Things has become the third wave of the information industry and cloud computing, big data, and Internet technologies. Among the many identification technologies used in the Internet of Things, radiofrequency identification technology is undoubtedly one of the most popular methods today. It is replacing the traditional contact IC card and becoming a new trend of smart cards. At the same time, a large amount of data is generated in the IoT environment. A lot of data involve user privacy, and users do not have good control over these data. Collecting and utilizing these data on the basis of protecting user privacy have become an important problem to be solved urgently. With the implementation of the strategy of rejuvenating the country through science and education, major colleges and universities are developing rapidly through enrollment and expansion, which also brings inconvenience to campus security management. Although the traditional campus all-in-one card system can guarantee the security identity of people entering and leaving, it does not reasonably integrate and utilize this information, resulting in waste of information resources and, to a certain extent, the problem of user privacy leakage. To solve the above problems, a new system was developed to integrate resources to identify users. To protect the privacy data of Internet of Things users, a specific solution using blockchain technology is proposed; for the identity authentication problem of Internet of Things users, the identity authentication based on the public key address of the blockchain is used on the chain, and the group signature is used off the chain. The identity authentication method solves the contradiction between anonymity and traceability in blockchain application scenarios. The simulation results show that the system not only considers user privacy but also has extremely important practical significance for the promotion of Internet of Things and RF applications.

## 1. Introduction

Recently, with the gradual miniaturization and intelligence of hardware components, the popularity of the IoT has become higher and higher, and it is involved in smart homes, electronic medical care, body area network, and Internet of Vehicles. The arrival of the 5G era will promote the IoT in thousands of households. Since the IoT system involves a large amount of user privacy information, protecting this privacy has become a key issue affecting the popularization of the IoT [1–3]. Because of the value of private data and the openness of the network environment, entities participating in the IoT may be subject to various types and degrees of external and internal attacks at any time. If private information cannot be protected, it will be difficult for users to accept this emerging technology, and the popularization of the IoT will be impossible. Therefore, the research on user privacy protection schemes in the IoT environment needs to continue to advance [4–6].

As one of the emerging technologies in recent years, the IoT has become more popular with the development of the economy and the improvement of living standards. In terms of home furnishing, people are looking forward to having an automated and intelligent home environment, such as moving target intrusion detection, gas leakage monitoring and alarming, temperature monitoring and automatic adjustment, and a series of electrical appliances that are automatically turned on and off according to the owner's living habits; in medical care, people hope to carry monitoring nodes with them, monitor the health of the human body, and automatically call medical assistance in case of emergency; in intelligent door locks, users do not need to carry keys after leaving and only need facial recognition or passwords to open the door locks. These ideas are nothing short of unrealistic in the past, and the emergence of 5G has made the Internet of Everything possible [7–9].

In a common IoT environment, entities can generally be divided into three types. One is the sensor node responsible for collecting data and executing received instructions; the other is the gateway node, which is responsible for uploading the data collected by the sensor node and sending it to the sensor node. It conveys the user's instructions and acts as a communication bridge; the last category is the user-side control terminal, which can summarize the entire system and perform a series of operations on its entities [10, 11]. Regardless of whether the user is within the scope of the system deployment or at a distance, he or she can control and monitor the system by communicating instructions to the gateway node after completing the authentication. In some special IoT environments, users are often in a state of high-speed movement, so frequent identity authentication is required, such as the Internet of Vehicles and air traffic control systems. Taking the Internet of Vehicles as an example, the entities in the Internet of Vehicles can be divided into three categories: users, vehicles, and roadside units. The vehicle is a special node that is always in a moving state and needs to continuously authenticate its identity to the RSU along the way [12–14].

While the IoT provides convenience for people, it also brings certain risks to users. The IoT involves a lot of user privacy, especially the monitoring and security modules and remote communication modules. Criminals can monitor the user's work and life by stealing the user's control terminal or directly invading the IoT system. The content of the user's communication may further commit the crime of extortion, theft, or robbery; steal the user's password to enter and leave the user's home at will; or forge the identity to steal the user's vehicle and resell it for illegal profit or use the vehicle to engage in illegal transportation activities in the name of the user. Once criminals exploit the IoT system, it will bring serious threats to the personal safety and property of users. Therefore, a reliable privacy protection solution plays a vital role in the IoT and is an essential factor in promoting the IoT's popularization [15–17].

Limited by hardware cost and software technology, the IoT was only developed within the military system in the early days of its existence. With the advancement of related technologies such as wireless sensor networks, electronic components, and the Internet, the IoT has gradually spread from a single military field to civil field, smart grid, body area network, digital medical care, smart home, Internet of Vehicles, and radiofrequency identification system, and they are all derived systems of the IoT [18, 19]. Through these IoT systems, users can operate machines without contact, observe and collect data remotely, receive system abnormal alarm information anytime and anywhere, and deal with them in time. The realization of all these functions is inseparable from the information interaction between entities. Information exchange in the IoT can be done through secret channels that are not open to the outside world, but in most cases, it is necessary to use open public channels to realize wireless communication [20–22]. At present, there are application environments in the IoT environment that require the intensive transmission of instructions, exchange of real-time information or continuous data collection, and frequent data transmission and message interaction, such as smart grid and smart home. Identity legitimacy checks are conducted without interacting with other messages or IoT systems that require short-length and low-frequency interaction messages, such as RFID systems, air traffic control systems, and identity information identification in the Internet of Vehicles. However, there are still some urgent problems to be solved in information security in the IoT application system. For example, in the Internet of Vehicles, users are required to directly use their real IDs to interact with other entities, which will expose the user's real-time location to the entire system. Any attacker can query the user's real-time location and travel trajectory as long as they invade the network and protect the user's private information [23–25].

This article mainly focuses on the protection of the privacy data of IoT users. The data generated by IoT users contain a large amount of personal privacy information. The unencrypted data are stored in the data center or cloud server. When the adversary obtains the data center's data, the user can be analyzed. Privacy behavior: the leakage of user privacy data will cause a series of user privacy leakage problems, which have great security risks. Adversaries easily forge the data files stored in the data center, and because the data center stores a large amount of data, it is difficult to detect when some data are forged or tampered with, and the tampered data are mixed with normal data for subsequent learning. Taking advantage of the immutability and decentralization of the blockchain, a blockchain-based IoT user privacy data protection scheme is proposed [26].

There are five sections in the article designed as follows: the first section introduces the origin of blockchain technology and IoT technology and the research status at home and abroad. The second section introduces the basic research of blockchain technology. The third section is the research on the privacy data protection of IoT users based on blockchain. The fourth section is the design and implementation of a blockchain-based IoT user privacy data protection scheme. In addition, according to our proposed blockchain-based IoT user privacy data protection scheme, the test scheme and test cases are determined, the function test and performance test of the system are carried out according to the test cases, and the test results are analyzed. The fifth section is the conclusion and outlook.

The research contributions of the study are as follows:

1. The study develops a new system to integrate resources to identify users.
2. The study proposes a specific solution using blockchain technology.
3. The study adopts the identity authentication based on the public key address of the blockchain, and the group signature is adopted off the chain. The identity authentication method solves the contradiction between anonymity and traceability in blockchain application scenarios.

## 2. Related Work

This study introduces the basic theory related to blockchain technology and the smart contracts, consensus mechanism, block structure, and group signature algorithm in the blockchain.

### 2.1. Peer-to-Peer Network

There is no central authority in a peer-to-peer network and is not bound by central system standards, so even if one peer in the network quits, you can still download from other peers.

The blockchain network is such a peer-to-peer network, as shown in Figure 1. Transactions and blocks in the blockchain are propagated between participating nodes through the blockchain network. The flooding algorithm in the blockchain network can ensure that data are in the network. It spreads quickly and can be stopped in time, without unlimited retweets. After the node in the Bitcoin blockchain receives the data, it will verify the transaction's validity. If it is valid, it will check whether it has been stored locally. If it has not been accepted, it will be stored locally and then forwarded to neighbor nodes; if received, it will not be forwarded.

### 2.2. Consensus Mechanism

A leader or board cannot make decisions in a blockchain of directors because blockchains have no “leaders.” In order for decisions to be made within the blockchain, consensus needs to be reached within the network using a “consensus mechanism.” In simple terms, consensus is a dynamic way of reaching a common agreement in a blockchain network, and reaching consensus ensures that trust in the blockchain is achieved for the benefit of the entire network. The more famous consensus mechanisms include workload proof mechanism, equity proof mechanism, and delegated equity proof mechanism with the following conditions:

(1) $$\begin{array}{c} \text{Conditions}\left(t\right)=\left\{\begin{array}{cc} \frac{2t-2t_{\min}}{t_{\max}-t_{\min}}, & t_{\min}\leq t\leq \frac{t_{\max}+t_{\min}}{2},\\ \frac{2t_{\max}-2t}{t_{\max}-t_{\min}}, & \frac{t_{\max}+t_{\min}}{2}\leq t\leq t_{\max},\\ 0, & t\leq t_{\min}\_\text{or}\_t>t_{\max}. \end{array}\right. \end{array}$$

The difficulty level of the puzzles will vary depending on the speed at which the blocks are mined. If the blocks are created quickly, then the puzzle will be more difficult and vice versa. Therefore, the puzzle's difficulty level must be adjusted in time to create a new block within a specific time frame. Several popular cryptocurrencies, such as Bitcoin, utilize a proof-of-work consensus mechanism. However, the rate of resource consumption by the proof-of-work consensus mechanism is particularly exaggerated, and this consensus mechanism wastes a lot of computing resources.

Proof of stake uses a random process to determine who has the power to produce the next block. Blockchain users can lock a portion of their assets for a certain period of time to become validators, and after becoming validators, users can generate blocks. Validators can also be selected based on the design of the blockchain. Generally, users with the largest stakes are more likely to gain the power to create new blocks.

Validators typically receive all or a portion of transaction fees for all transactions made in blocks they create, or, alternatively, validators may receive a specific amount of currency due to inflation. In this way, the proof-of-stake method can incentivize validators to maintain the blockchain network. Proof of stake saves computing resources compared with other blockchain consensus mechanisms such as proof of work [25].

### 2.3. Cryptography

One of the most fundamental goals of cryptography is to enable parties to communicate through open communication channels in a secure manner. Secure communication means guaranteeing the confidentiality and verifiable integrity of the message. Confidentiality prevents an adversary from learning any information about the content of the message. Integrity requires that each party should be able to identify whether the received message was sent by the claimant. One party of the message was sent, and the message was not tampered with in transit, including the source of the message and the content of the message [26].

Typical private key encryption algorithms are DES, AES, etc. Although the encryption scheme can be implemented correctly, there are some inherent disadvantages: the sender and receiver must share the same public key; it is difficult to implement in many cases, such as in the Internet middle.

Public key encryption, also known as asymmetric encryption, solves the problem of the difficulty of key distribution in private key encryption. The receiver B has a key pair: public key and private key. The public key is published so that everyone knows it, while B stores the private key secretly, others use B's public key to encrypt the emails sent to B, and only B can use his private key to decrypt them, thereby securely communicating.

The public key encryption scheme also consists of three probabilistic polynomial time algorithms: KeyGen, Encrypt, and Decrypt.

(2) $$\begin{array}{c} \text{KeyGen}\left(\right)=\left(pk,sk\right). \end{array}$$

The key generation algorithm KeyGen generates a public-private key pair (*pk*, *SK*).

(3) $$\begin{array}{c} \text{Enc}\left(pk,m\right)⟶\sigma . \end{array}$$

The encryption algorithm Enc takes the public key *pk* and the message *m* as input and outputs the ciphertext result.

(4) $$\begin{array}{c} \text{Dec}\left(sk,c\right)⟶m. \end{array}$$

The decryption algorithm Dec takes the private key *SK* and the ciphertext as input and outputs the plaintext *m*.

(5) $$\begin{array}{c} \text{Dec}\left(sk,\text{Enc}\left(pk,m\right)\right)⟶m. \end{array}$$

Private key encryption schemes (KeyGen, Encrypt, Decrypt) must satisfy the following correctness requirements: any key pair (*pk*, *SK*) and any message *m* output by KeyGen() meet the requirement as formula (4).

## 3. Research on IoT Privacy Data Protection Scheme

### 3.1. IoT User Authentication Problem

Blockchain-based IoT user privacy data protection first considers the identity authentication of IoT users. Blockchain is an authentication method based on public key addresses. Users in the network have a one-to-many relationship with public key addresses. Users' privacy is guaranteed under the protection of this pseudo-anonymity. However, research shows that the pseudo-anonymity of the blockchain cannot eliminate the risk of privacy leakage. It is beneficial to trace the source of the problem, so an improved authentication scheme that can balance anonymity and traceability problems is needed.

(6) $$\begin{array}{c} \min F_{\text{obj}}=\min P+\lambda {\sum_{\beta }\left[\frac{V_{i}-V_{i\lim}}{V_{i\max}-V_{i\min}}\right]}^{2}. \end{array}$$

Blockchain can be used as authentication, and users register their identity on the blockchain using their key pair. This registered identity is information that contains a hash of several identity-related attributes. Afterward, such users can join a recognized group that verifies the hashes registered earlier on the blockchain and then have the identifying party confirm that information as truth on the blockchain. Other parties who trust a particular identified party can now trust the identity on the blockchain and use it as an authentication or identification mechanism, but users may lose their identification, for example, the loss of a cell phone or other data carrier that stores the private key portion of an identity, or even worse: data theft of a digital identity. In the case of decentralized authentication based on blockchain technology, no central entity controls the identity where a new identity can be requested and my old identity marked as stolen or lost in the blockchain. In another case, since the blockchain provides pseudo-anonymity, everyone corresponds to one or more public key addresses on the blockchain, that is, a virtual identity, although having multiple public key addresses can enhance the anonymity. However, studies have shown that when on-chain transactions are linked with off-chain, the real identity behind the virtual identity can be revealed by analyzing a large amount of transaction data, thereby exposing user privacy.

(7) $$\begin{array}{c} \theta^{e+1}=\theta^{e}+\frac{\alpha }{\left|B\right|}{\left(X^{B}\right)}^{T}\left(X^{B}\theta^{e}-y^{B}\right). \end{array}$$

We provide IoT users with public and private key pairs based on the Ethereum blockchain technology. Data are only considered valid data in the case of valid blockchain signatures and group signatures. If malicious users send data to the block at will, the chain can destroy the system's stability, and the signer can be traced through the private key of a specific group manager for punishment. Since the blockchain technology itself does not have the traceability feature, it cannot effectively punish malicious users who destroy the system's stability. The traceability feature of the group signature just makes up for this defect and guarantees the effective management of the system. It is shown in Figure 2.

### 3.2. User Privacy Data Integrity Verification Problem

After introducing the identity authentication of IoT users and the storage method of IoT user privacy data, we mainly analyze the integrity verification of IoT user privacy data and how to ensure user privacy, and the detailed work flow chart is shown in Figure 3.

**Step 1 .**

The IoT user joins the user group to obtain the private key of the group members, uploads the data to be uploaded to IPFS, and obtains the returned data content address (hash value).

(8) $$\begin{array}{c} {\hat{x}}^{\left(0\right)}\left(k+1\right)={\hat{x}}^{\left(1\right)}\left(k+1\right)-{\hat{x}}^{\left(1\right)}\left(k\right). \end{array}$$

**Step 2 .**

The IoT user invokes the group signature algorithm and the Ethereum digital signature algorithm to calculate the group signature and the elliptic curve digital signature, respectively.

(9) $$\begin{array}{c} {\hat{x}}^{\left(0\right)}\left(k+1\right)=\left({\hat{x}}^{\left(0\right)}\left(1\right)-\frac{b}{a}\right)e^{ak}+\frac{b}{a}. \end{array}$$

**Step 3 .**

The IoT user calls the set() function in the smart contract to upload the data identification. The smart contract verifies whether the sender himself signs the digital signature. If the signature is correct, the data identification will be uploaded to the chain; if the signature is incorrect, upload operations are retuned before the data.

(10) $$\begin{array}{c} {\hat{x}}^{\left(0\right)}\left(k\right)+{\hat{ax}}^{\left(1\right)}\left(k+1\right)=b. \end{array}$$

**Step 4 .**

Other users in the system call the get() function in the smart contract to obtain the user data of the specified group ID.

**Step 5 .**

According to the group ID and group signature in the obtained data identification, the correctness of the group signature is verified through the group signature server. If the verification is correct, the next step is proceeded. If the verification fails, the corresponding group administrator is reported to track the signature and upload error. Group signers of the information take corresponding punitive measures.

(11) $$\begin{array}{c} ab=\left(a_{1}+\cdots +a_{n}\right)\left(b_{1}+\cdots +b_{n}\right)=\sum_{i=1}^{n}\sum_{j=1}^{n}a_{i}b_{j}. \end{array}$$

**Step 6 .**

Data are obtained from IPFS according to the data content address in the data identifier, the correctness of the data hash is verified locally; if it is correct, the integrity verification is completed; if the verification is incorrect, the next step is proceeded where the verification fails in Step 5.

(12) $$\begin{array}{c} \Delta X_{t}=\alpha +\beta_{t}+\gamma X_{t-1}+\sum_{i=1}^{m}\beta_{i}\Delta X_{t-i}+\sum_{i=1}^{m}\beta_{i}\Delta X_{t-i}. \end{array}$$

### 3.3. User Privacy Data Storage Issues

In the IoT environment with frequent identity authentication, such as the Internet of Vehicles and air traffic control systems , users are often in a state of high-speed movement, and they need to frequently conduct identity authentication to fixed authentication nodes along the way. The system has extremely high requirements for the timeliness of authentication information. Therefore, the protocol design needs to simplify the authentication steps as much as possible and improve authentication efficiency to protect user privacy. Because the authentication factor may be stolen, the reliability of the authentication mechanism relying on a single factor is weak. Based on this, this study proposes a multifactor-based lightweight anonymous authentication protocol for this special IoT environment to meet the needs of frequent system authentication.

(13) $$\begin{array}{c} \left\{\begin{array}{c} V_{\min}\leq V_{i}\leq V_{i\max},i\in N_{PV},\\ T_{k\min}\leq T_{k}\leq T_{k\max},k\in N_{T},\\ Q_{c\min}\leq Q_{Ci}\leq Q_{c\max},i\in N_{C},\\ V_{i\min}\leq V_{i}\leq V_{i\max},i\in N_{PQ},\\ P_{Gi\min}\leq P_{Gi}\leq P_{Gi\max},i\in \left\{N_{PV},S\right\}. \end{array}\right. \end{array}$$

This protocol uses authentication factors such as smart cards and biometric templates to simplify some authentication processes and provide a fast and efficient authentication method for legitimate users who have been authenticated once while improving the authentication efficiency.

It strengthens the protocol's reliability and guarantees the privacy protection of users. In the multifactor-based lightweight anonymous identity authentication protocol proposed in this study, the user needs to first input the personal biometric template to verify the identity legitimacy of the mobile device and then only needs to perform a complete calculation to the nearest authentication node during the first authentication operation, and you can use the parameters obtained from the initial authentication to more easily complete the subsequent identity authentication to the authentication nodes along the way, which is shown in Figure 4.

## 4. Experimental Result Analysis

Figure 5 shows the changing trend of the successful probability of attack node fork attack tampering followed by the number of blocks *z*. The three curves represent the ratio of honest node computing power *p* to attack node computing power *q*: 10 : 1, 9 : 3, and 7 : 3. It can be seen from the figure that when the computing power of honest nodes accounts for the majority, as the number of subsequent blocks increases, the probability of blocks being tampered with decreases exponentially, and the greater the proportion of computing power of honest nodes, the faster the confirmation speed.

The time consumption comparison is shown in Figure 6. The call time consumption of each function is an average of 30 calls. It can be seen from the figure that the overall function call time of the remote virtual machine is higher than that of the local call time. The request function with the highest time consumption is the group 1 function as shown in (8), which is 0.32 s and 0.24 s, respectively, followed by the group 5, group 4, and group 3 functions, which are defined as equations (9), (10), and (12), respectively. The actual computational complexity is consistent, and the overall time consumption is within an acceptable range.

According to the survey results in Table 1, our proposed scheme can prevent putative attacks based on efficiently storing data compared with other blockchain-based schemes. Compared with other methods, our method can prevent data tampering without revealing user privacy, IoT users have ownership of data, and supporting smart contracts means that the system has more room for improvement. In the table, “Y” and “N” indicate satisfaction and dissatisfaction, respectively, “L” indicates that the scheme has certain performance defects, “H” indicates that the scheme is efficient, and “M” indicates that the method is feasible; still, there is room for improvement.

## 5. Conclusion

To solve the problem of user privacy protection information security, this study designs two secure communication protocols for different IoT environments that operate frequently: a multifactor-based certificateless signcryption protocol and a multifactor-based lightweight anonymous authentication protocol. Both schemes provide message confidentiality and integrity and protect user privacy during communication. They provide a secure foundation for other applications in an IoT environment. The main work of this study is summarized as follows: first, for the IoT environment with frequent message exchange, a multifactor-based certificateless signcryption protocol is proposed. The protocol computes and uses biometric keys to strengthen the authenticity and legitimacy of verifying the user's identity. Then, for the IoT environment where identities are frequently authenticated, a multifactor-based lightweight anonymous authentication protocol is proposed. In this protocol, only the registration authority has the corresponding relationship between the user's real identity and pseudo-identity and supports anonymous and traceable identity authentication.

Although this study proposes a blockchain-based privacy data protection scheme, there are still many issues to be considered in terms of the efficiency and storage capacity of smart contracts. The value of blockchain technology in protecting user privacy is unquestionable. However, to truly integrate into the IoT scenario, there is still a lot of room for improvement. The speed of block generation and the appropriate consensus mechanism are the key points and difficulties that need to be studied.

## Figures and Tables

**Figure 1:** Peer-to-peer networks and the C-B model.

**Figure 2:** IoT user authentication.

**Figure 3:** Blockchain-based IoT user privacy data integrity verification process.

**Figure 4:** IoT system framework for frequently authenticated identities.

**Figure 5:** Attack node fork success probability.

**Figure 6:** Group signature service time consumption.

**Table 1:** Performance on different aspects of IoT.

Group	Fraud prevention	Tamper proof	Traceability	Anti-replay
1	Y	47.2	0.82	H
2	Y	55.3	0.92	H
3	Y	50.5	0.84	L
4	N	58.3	0.92	L
5	N	52.2	0.82	M
6	N	61.2	0.92	M
7	N	62.1	0.94	H
8	N	55.6	0.82	L
9	Y	65.9	0.94	L
10	Y	79.0	0.91	M
11	N	60.3	0.82	M
12	Y	75.4	0.94	H
13	N	78.7	0.74	111.5

## Data Availability

The data used to support the findings of this study are available from the corresponding author upon request.
